RETRACTED

# A multiple information model incorporating limited attention and information environment

**DOI:** 10.1371/journal.pone.0257844

**Published:** 2021-10-07

**Authors:** Tong Chen, Ziqing Chen, Xuejun Jin

**Affiliations:** School of Economics, Zhejiang University, Hangzhou, China; Ministry of Natural Resources North Sea Bureau, CHINA

## Abstract

Rapid development of intelligent information equipment accelerates the expansion of mobile social network. Speed of information spreading is gradually growing, there are lots of changes in the scale and mode of information spreading. But the basic communication network is not developed and not mature, when online information platforms breakdown sometimes it happens to be when important information appears. Therefore, the research is done to solve these occasion problems, help network information platform filter hot news and discuss the reason that hot news exists longer than other news in the Internet. In this paper, a multiple information propagation model incorporating both local information environment and people’s limited attention is proposed based on Susceptible Infected Recovered (SIR) model. Two new concepts are introduced into the model: heat rate and popular rate, to measure the local information influence power and people’s limited attention to information respectively, which are key factors determining node state transformation instead of fixed probability. In order to analyze the influence from limited attention, a situation is designed that several pieces of information are popular successively. The theoretical analysis shows that the early popular information gets more attention than the later popular information, and more attention makes it easier to spread. Besides, numerical simulation is conducted in both uniform network and scale-free network. The simulation results show that the early popular information is less vulnerable to the increase of information acceptance threshold and more sensitive to the decrease of information rejection threshold than the later popular information. Moreover, the model can also be used in the case of large amount of information transmission without adding too much complexity. Reasons are given in the research that the top hot news exists very much longer than the other ones, and latter news which have same influence as top news are hard to get the same focus. Meanwhile, results in the research can provide some ways for the other researches in the related fields. They also help related information platforms to filter and push news and referable strategies to maintain hot news.

## 1. Introduction

With the development of Internet and social media, people are living in an environment of information explosion. Social media have greatly changed the way of information release and dissemination. People often face multiple information during a period of time, but their attention is limited. When multiple information spreading in a social network, how these pieces of information interact with each other and how people’s attention affects information propagation are worth studying. It is often seen that online platform breaks down due to the heavy burdens on webserver when an important message is needed to be sent to all users through online information platform but massive users are searching related information by themselves. Besides, users are easy to be distracted by unnecessary information, which cause that important messages cannot be conveyed to all the users in need immediately. Scheme in the research can help online information platforms lighten the burdens to avoid that situation, divide and filter useful information for users, and make information spreading more effective.

RETRACTED

There are a lot of studies on information propagation in social network. Early research focused on single information propagation, and some epidemic models, such as susceptible-infective-susceptible (SIS) model [1,2], susceptible-infective-removed (SIR) model [3,4] and susceptible-exposed-infective-removed (SEIR) model [5,6], were used to describe the information propagation in social network. These models were analyzed in both homogeneous and heterogeneous social networks [7–10]. In the real world, there is often multiple information spreading during a period of time, so the analysis of multiple information dissemination has begun to be the focus of research recently. Previous studies have demonstrated that the interaction among different pieces of information is either cooperation or competition. Some researchers suppose that a node can only transmit a piece of information when competitive information spreading in a social network [11–13], while others assume that a node can be infected by multiple information at the same time during the information propagation process [14,15]. Besides, the situation that one piece of information unilaterally inhibits the other is also analyzed, for example, Huo and Song (2016) proposed a model in which rumor and scientific knowledge are simultaneously spreading in a system and the spreading of scientific knowledge can prevent rumor diffusion [13]. In addition, some scholars have proposed another model by adding new hesitators as a neutral state of dual information competition, where both hesitators and spreaders can facilitate the information dissemination [14].

The above studies focused on multiple information propagation in single layer network, while other researchers studying multiple information spreading in multiplex networks. In multiplex networks, the nodes are overlapped with several interconnected sub-networks. Li et al. (2019) revealed the diffusion process of mutual promotion and restraint between multiple information and they introduced a dynamic interaction mechanism based on the multiple SIS diffusion model [15]. Xiao et al. (2019) proposed the MM-SIS (multiple information and multiplex network SIS) model to analyze the interaction between different information and different propagation paths [16]. He and Liu (2020) proposed a competitive information dissemination model, and they analyzed the competition mechanism and the information propagation evolution laws according to Markov chain theory [17]. Ivokhin et al. (2018) proposed a model incorporating dynamics and mathematics to formulate the process of information spreading in people from a specific society or area [18]. Srivastava and Sankar (2020) put forward a new method to identify errors under throwable in the server of online information platform and conduct a predicting survey on the social data of Twitter (online social platform) under extreme weathers. Then qualitive analyses can be made on the data collected from social media and website of weather information [19]. Tulu et al. (2018) proposed condition-based Maintenance (CbM), which measured entropy that randomly moves between nodes and neighbors. Method of CbM described the importance of nodes being connected to two or more online neighbors. Relativities were discussed between CbM and other classic methods of identifying influential nodes are [20].

RETRACTED

Although the prior work has made considerable achievements, there are still some limitations: First, all the multiple information propagation models are based on pairwise information interaction, so the models will be very complex if the amount of information is too large. Therefore, these models are difficult to be extended. Second, the transformation among different node states is usually set as a fixed probability, and the important local information environment is ignored. Third, most of the previous models suppose multiple information transmits simultaneously while the situation of multiple information arriving successively is ignored.

In this paper, another multi-information model is proposed in which a node’s state is largely affected by its surrounding neighbors’ states and people’s limited attention plays a key role in the interaction of multiple information. The nodes’ psychological characteristics, such as hesitation and forgetting [21], herd behavior [22,23] and risk averse thoughts [24,25], are internal factors influencing information spreading process in social networks and have been analyzed. The Ising model [26–28] and its extended models [29,30] are often used to explain the herd effect and the opinion evolution process, and according to these models, people’s opinions are largely affected by their neighbors’ opinions. Inspired by psychological studies and the Ising model, people’s limited attention and the states of nodes’ neighbors as key factors are considered in the multiple information spreading model. People’s attention is limited and distracted [31–33], and it can be easily attracted by hot spots, when someone is interested in one thing, one’s attention will be reduced in other events. Moreover, here is an assumption that the early coming information has more exposure than latter one, and the order of information can influence the information dissemination effect.

RETRACTED

The main contributions of this paper are as follows:

1. Proposal of a new multi-information propagation model in which both local information environment and limited attention are introduced as the determinant factors of node state transformation, instead of initial setting fixed probability as other models do.
2. The model is also suited to the situation where there is a vast amount of information transmitting because this model will not get extremely complex in that case as other models. These methods have good reference value for other models.
3. A situation is designed, where multiple information arrives successively, which is different from multiple information spreading simultaneously in previous studies. Therefore, this model can be used to explain the order effect of information on the information propagation process.

The rest of this paper is organized as follows. Section 2 introduces this multi-information propagation model in detail. Section 3 shows the theoretical analysis of this model. Section 4 analyzes this model in simulation method, the analysis in both uniform network and scale-free network are included. Finally, section 5 concludes all this paper.

## 2. Multi-information propagation model

In this section, multi-information spreading model is introduced in detail. The model is based on classic Susceptible Infected Recovered (SIR) epidemic model [3,4]. In this model, a population of *N* individuals is divided into three states: susceptible (*S*), infective (*I*) and removed (*R*). “*S*” represents the people who do not know the information, “*I*” represents the people who have been affected by this information and they can spread this information to *S* group. “*R*” represents the people who have heard the information but do not agree with this information. What’s more, *R* also encourages other group members to join in *R* group, but *R* will not transform to other states anymore.

RETRACTED

According to this classic spreading model, the total population size is represented as *N* (*N* is constant), and *S(t)*, *I(t)*, *R(t)* represent the fraction of nodes which are in the susceptible, infective and removed states, respectively, and *S(t)*, *I(t)*, *R(t)* will change as time *t* goes by due to the interactions among these groups. The sum of these fractions equals to 1:

S(t)+I(t)+R(t)=1 (1)

In Eq (1), *S(t)* represents the susceptible; *I(t)* represents the infected; and *R(t)* represents the removed states. Inspired by the Ising model [26–28], the information environment is supposed to have a large influence on one’s acceptance of information, and in the model, “temperature” is defined as *T* and “heat rate” is defined as *H* to quantify this influence. For all the information, *T* represents the average influence power from one’s all neighbors:

$$T=\sum_{i}^{n}d_{i}/n$$ (2)

In Eq (2), *T* represents the temperature; and *H* represents “heat rate”, where *d*_*i*_ represents the degree of personal influence and *n* represents the quantity of neighbors of a user. The degree of personal influence means the impact of oneself, here the degree is defined as one’s connection link number with one’s neighbors.

In the model, another concept “heat rate” *H* represents the sum of one node’s neighbors’ attitude divided by average influence power of all neighbors, and it reflects the information influence power on this node.


$$H=\sum_{i}^{n}a_{i}∙d_{i}/T$$ (3)

In Eq (3), *a*_*i*_ represents the attitude of user “*i*”. and $\sum_{i}^{n}a_{i}∙d_{i}$ represents the sum of a node’s neighbors’ attitude. Here the attitude of *S* is represented as *a*_*S*_, equaling to 0, which means the attitude of *S* neighbor has no effect on the selected node. Besides, the attitude of group *I* and *R* is defined as *a*_*I*_ and *a*_*R*_, and set as 1 and -1, respectively. The attitudes of group *R* and *I* are set as absolute equal value because they are considered to have the same influence power for the information receiver, no matter the receiver is in attitude *S*, *I* or *R*. The influence power is mostly determined by the spreading person, which has been defined as degree *d*_*i*_. $\sum_{i}^{n}a_{i}∙d_{i}$ also shows that the attitudes of group *I* and *R* can offset each other, which is reasonable because many different and opposite attitudes of one information can confuse one person, so here the attitude with the larger absolute value is simply considered to have a greater impact.

RETRACTED

The value of *H* equals to the sum of neighbors’ attitude over the average influence degree *T*, so it can be large if one’s neighbors are mostly hold *I* or *R* attitude, and it will be small if the number of *I* and *R* is close or most of the neighbors hold *S* attitude.

Since *H* can be very large, it is transformed into a limited range on. Here the general activation function is used:

τ=tanh(H) (4)

In Eq (4), *τ* represents the quantity of nodes in the conversion and the final judgement index. The evolution tendency of function (4) is shown in Fig 1, and it can be seen that the value of *τ* will be closer to 1 when *H* gets larger, and it will be closer to -1 when *H* gets smaller.

**Fig 1:** The evolution tendency of *τ* with H changing from negative to positive.

Here the method is introduced that is used to deal with the multi-information situation. The absolute value of one’s attitude is used, in order to reflect the attention degree of chosen information, like:

$$A=\sum_{i}^{n}\sum_{j}^{m}|a_{ij}|∙d_{i}$$ (5)

In Eq (5), *A* represents the degree how all users focus on all information nodes, and *a*_*ij*_ represents the degree of attention of user *i* on the information *j*. Similarly, the attention degree can be defined as *A*_*j*_ for information *j*:

$$A_{j}=\sum_{i}^{n}|a_{ij}|∙d_{i}$$ (6)

In Eq (6), *A*_*j*_ represents the degree of all users’ attention on the information *j*. Absolute attitude value is used in the calculation of *A*_*j*_, because although the node with *R* statement holds the different views or holds the prudent views, the attention of this node is still attracted by this information.

Similar to Eq (2), the “popular temperature” can be used for information:

$$TI=A/m=\sum_{j}^{m}A_{j}/m$$ (7)

In Eq (7), *TI* represents average degree of population in all information. And, the “popular rate” can also be defined for information *j*:

$${\mathrm{HI}}_{j}=A_{j}/TI$$ (8)

In Eq (8), *HI*_*j*_ represents the average degree of population of information *j*, and in general, larger *HI*_*j*_ means information *j* can attract more attention. Since *HI*_*j*_ can also be very large, the same method is used, activation function tanh(), to transform *HI*_*j*_ into range (0, 1), where *HI*_*j*_∈[0, +∞), tanh(*HI*_*j*_)∈[0, 1).

The heat rate *H* is combined with *HI* to get the final judgement parameter *J*_*j*_:

$$J_{j}=\tau_{j}\tanh\left({HI}_{j}\right)=\tanh\left(H_{j}\right)\tanh\left({HI}_{j}\right)=\tanh\left(\frac{\sum_{i}^{n}a_{ij}∙d_{i}}{\sum_{i}^{n}d_{i}/n}\right)\tanh\left(\frac{\sum_{i}^{n}|a_{ij}|∙d_{i}}{\sum_{j}^{m}\sum_{i}^{n}|a_{ij}|∙d_{i}/m}\right)$$ (9)

where larger *HI*_*j*_ will make *J*_*j*_ become closer to original *τ*_*j*_, while smaller *HI*_*j*_ will make *τ*_*j*_ lose influence and make *J*_*j*_ become closer to 0.

RETRACTED

After getting the value of *J*, α,β,γ,η are used to determine the possible transformation between different groups. The transformation result is based on the calculated value *J*, the selected node and the connected node. Here *c*_*A*_ is used to represent the selected node, and *c*_*B*_ is used to represent the connected node. The connect probability is based on the degree of person himself. It is more likely that *c*_*A*_ chooses a large degree neighbor to connect, here the node pick probability is set to equal to each neighbor’s degree over the sum of all neighbors’ degree.

All the transformation cases for the selected node are as follows:

1. *c*_*A*_ = *S*, *c*_*B*_ = *I*, *J*≥α_0_: *c*_*A*_ transforms to *I*, *c*_*A*_ = *I*;
2. *c*_*A*_ = *I*, *c*_*B*_ = *R*, *J*≤β_0_: *c*_*A*_ transforms to *R*, *c*_*A*_ = *R*;
3. *c*_*A*_ = *S*, *c*_*B*_ = *R*, *J*≤γ_0_: *c*_*A*_ transforms to *R*, *c*_*A*_ = *R*;
4. *c*_*A*_ = *I*, *J*≤η_0_: *c*_*A*_ transforms to *R*, *c*_*A*_ = *R*;
5. *c*_*A*_ = *R*: *c*_*A*_ does not transform.

Here α_0_, β_0_, γ_0_ represent the threshold of transformation from *S* to *I*, *I* to *R* and *S* to *R*, respectively, while *η*_0_ represents the threshold of transformation from *I* to *R* by the environment influence. The threshold means when the environment situation meets the condition, such as *J*≤β_0_, then the transform parameter is set as β = 1, otherwise β = 0. The other parameters α, γ, η also follow this regular.

In this model the attitude value of *I* and *R* are set to equal to 1 and -1 respectively, so if the neighbors’ attitude is close to *I*, the value of *τ* should be close to 1, and this is the reason why the judgement condition is set as *J*≥α_0_ in case 1. While if the neighbors’ attitude is close to *R*, the value of *τ* should be very close to -1, and the judgement condition should be *J*≤β_0_ (*J*≤γ_0_) in case 2(3). In case 4, it is supposed if the judgement parameter is very extreme and most of the node’s neighbors belong to *R* group, the node will change his mind from *I* to *R* automatically.

Since all the parameters depend on the local circumstance, based on the introduced details above, the local dynamic system can be written as:

$$\frac{ds(t)}{dt}=-\alpha s(t)i(t)-\gamma s(t)r(t)$$ (10)

$$\frac{di(t)}{dt}=\alpha s(t)i(t)-\beta i(t)r(t)-\eta i(t)$$ (11)

$$\frac{dr(t)}{dt}=\gamma s(t)r(t)+\beta i(t)r(t)+\eta i(t)$$ (12)

In Eqs (10–12), s(t), i(t) and r(t) respectively represent partial occupancy rate, compared with S(t), I(t) and R(t).

The process of judgement and the dynamic relationship between these groups are shown in Fig 2.

RETRACTED

**Fig 2:** The transformation model and dynamic relationship between different groups of the multi-information system.

## 3. The theoretical analysis

### 3.1 The equilibrium analysis

In order to analyze the equilibrium of this multi-information propagation system, the traditional method is to let Eqs (10)–(12) equal to zero. The results are easy to get as:

$$s(t)=\left(\alpha \beta +\alpha \eta -\gamma \eta \right)/\left(\alpha^{2}+\alpha \beta -\alpha \gamma \right)$$ (13)

$$i(t)=\gamma (\eta -\alpha )/\left(\alpha^{2}+\alpha \beta -\alpha \gamma \right)$$ (14)

r(t)=(α−η)/(α+β−γ) (15)

Since all the parameters in these equations depend on the local judgement *J*, these steady equilibrium results are suitable for local situation.

Besides, in the system α determines the spreading speed from group *S* to group *I*, Eq (14) can be transformed into:

$$\alpha =\frac{-\left[\beta i(t)-\gamma i(t)+\gamma \right]+\sqrt{{\left[\beta i(t)-\gamma i(t)+\gamma \right]}^{2}+4i(t)\gamma \eta }}{2i(t)}$$ (16)

Since in the system when *J* < α_0_, α = 0, so the stop spreading condition from group *S* to *I* is:

$$\alpha_{0}>\frac{-\left[\beta i(t)-\gamma i(t)+\gamma \right]+\sqrt{{\left[\beta i(t)-\gamma i(t)+\gamma \right]}^{2}+4i(t)\gamma \eta }}{2i(t)}$$ (17)

From the above assumption, the condition of group *I* local peak value can be gotten when only the spreading parameter α is changed:

$$i(t)<\gamma (\eta -\alpha_{0})/\left(\alpha_{0}^{2}+\alpha_{0}\beta -\alpha_{0}\gamma \right)$$ (18)

When the density (group occupancy in local area) of group *I* reaches this theoretical peak value, the spreading channel from *S* to *I* will be closed. Since the peak value of *I* depends on many parameters as mentioned above, the results in real situation will be more complex.

In this multi-information propagation system, all the transformations are based on the local judgement parameter *J*, so it is necessary to analyze its formation in detail to understand the changing tendency of this system.

### 3.2 Uniform network analysis

First, the case in uniform social network is analyzed. The derivative of *J* is:

$$J^{\prime }=H^{\prime }[1-\tanh^{2}\left(H\right)]\tanh\left(HI\right)+HI^{\prime }\tanh\left(H\right)[1-\tanh^{2}\left(HI\right)]$$ (19)

The results of *H* and *HI* depend on the local distribution of *S*, *I*, *R* as well as the structure of propagation network. Based on Eqs (2) and (3), in uniform network *H* can be rewritten as

$$H=n(i_{j}-r_{j})$$ (20)

In Eq (20), n represents the quantity of neighbors of selected node, where *i*_*j*_ and *r*_*j*_ respectively represent densities of *I* and *R* of information *j* around nodes. Similarly, *HI* can be rewritten from Eqs (5)–(8) as

$$HI=\left(i_{j}+r_{j}\right)/\left(\bar{i}+\bar{r}\right)=u(i_{j}+r_{j})$$ (21)

where $\bar{i}$ and $\bar{r}$ represent the average density from the surrounding nodes of all the information, and they can be written as:

$$\bar{i}=\sum_{j}^{m}i_{j}/m,\bar{r}=\sum_{j}^{m}r_{j}/m$$ (22)

And in $u=1/\left(\bar{i}+\bar{r}\right)$, *u* is used as a simplified parameter in Eq (21). The parameter *u* can be considered as the attention rate: small *u* means the surrounding nodes have received much information and will be hard to be interested in new information, while large *u* means the surrounding nodes are most in *S* state and easy to accept new coming information.

RETRACTED

It is easy to understand that $i_{j},r_{j},\bar{i},\bar{r}>0$ since the density of different groups cannot be lower than 0, and for the same reason we can get *n*, *u* > 0. In this situation, Eq (9) can be rewritten as

$$J=\tanh\left[n(i_{j}-r_{j})\right]\tanh\left[u(i_{j}+r_{j})\right]$$ (23)

Correspondingly, these are the derivatives of *J* for all the depending parameters.


$${J|}_{i_{j}}=n\{1-\tanh^{2}\left[n(i_{j}-r_{j})\right]\}\tanh\left[u(i_{j}+r_{j})\right]+utanh[n(i_{j}-r_{j})]\{1-{tanh}^{2}[u(i_{j}+r_{j})]\}$$ (24)

$${J|}_{r_{j}}=-n\{1-\tanh^{2}\left[n(i_{j}-r_{j})\right]\}\tanh\left[u(i_{j}+r_{j})\right]+u\tanh[n(i_{j}-r_{j})]\{1-{tanh}^{2}[u(i_{j}+r_{j})]\}$$ (25)

$${J|}_{n}=(i_{j}-r_{j})\{1-\tanh^{2}\left[n(i_{j}-r_{j})\right]\}\tanh\left[u(i_{j}+r_{j})\right]$$ (26)

$${J|}_{k}=(i_{j}+r_{j})\tanh\left[n(i_{j}-r_{j})\right]\{1-\tanh^{2}\left[u(i_{j}+r_{j})\right]\}$$ (27)

Now Eqs (24)–(27) are set to equal to zero, considered their second derivative to analyze the peak value conditions of *J* from these corresponding parameters.

For Eqs (26) and (27), it is easy to find the maximum and minimum condition for parameter *n* and *u* is *i*_*j*_ *= r*_*j*_, and only under that situation the steady value is *J* = 0. When *i*_*j*_ ≠ *r*_*j*_, *J* tends to be monotonic increasing (*i*_*j*_ > *r*_*j*_) or decreasing (*i*_*j*_ < *r*_*j*_).

Solving Eqs (24) and (25) in analytical approach are very hard since they are transcendental equations, here numerical calculation method is used to analysis this problem. Figs 3–5 show the change tendency of *J* and $J{|}_{i_{j}}$ with *n* = 2, *n* = 6 and *n* = 14, respectively. Combined with these three figures, it is found that the maximum of $J{|}_{i_{j}}$ is around *i*_*j*_ = *r*_*j*_, and with the increase of *n* and *u*, the appear position of maximum peak value is closer to the line *i*_*j*_ = *r*_*j*_, and the maximum of $J{|}_{i_{j}}$ also gets larger. Besides, the increase of *n* and *u* also lead to larger $J{|}_{i_{j}}$ peak value, leading to *J* reaches the upper peak value faster, and the maximum value of *J* is extremely depended on the value *n* and *u*. It is easily found that smaller *n* and *u* make *J* reach smaller peak value, means under the same condition, fewer neighbors and the larger other information occupancy will restrain the information spreading. Besides, small *n* will make *J* with no minimum point, and under that condition *J* also cannot reach a high value (Fig 3(A)–3(C)).

RETRACTED

**Fig 3:** The change tendency of *J* and $J{|}_{i_{j}}$ with fixing parameter *n* = 2. (a)–(c) shows the change of $J{|}_{i_{j}}$ by different *i*_*j*_ and *u* with *r*_*j*_ = 0.05, 0.20, 0.35, respectively. While (d)–(f) shows the change of *J* by different *i*_*j*_ and *u* with *r*_*j*_ = 0.05, 0.20, 0.35, respectively.

**Fig 4:** The change tendency of *J* and $J{|}_{i_{j}}$ with fixing parameter *n* = 6. (a)–(c) shows the change of $J{|}_{i_{j}}$ by different *i*_*j*_ and *u* with *r*_*j*_ = 0.05, 0.20, 0.35, respectively. While (d)–(f) shows the change of *J* by different *i*_*j*_ and *u* with *r*_*j*_ = 0.05, 0.20, 0.35, respectively.

**Fig 5:** The change tendency of *J* and $J{|}_{i_{j}}$ with fixing parameter *n* = 14. (a)–(c) shows the change of $J{|}_{i_{j}}$ by different *i*_*j*_ and *u* with *r*_*j*_ = 0.05, 0.20, 0.35, respectively. While (d)–(f) shows the change of *J* by different *i*_*j*_ and *u* with *r*_*j*_ = 0.05, 0.20, 0.35, respectively.

Due to the symmetry properties in this system, group *I* and *R* have the same strength of impact on judgement *J* but with totally different effect, so the results for $J{|}_{r_{j}}$ are just in completely opposite. Due to the limitation of space, the analysis for $J{|}_{r_{j}}$ will not be repeated here again.

### 3.3 Scale-free network analysis

Here are analyses of the situation in non-uniform social network. The traditional scale-free, or says BA network [34,35] has the degree distribution as:

$$P(k)=\frac{2m^{2}t}{m_{0}+t}\frac{1}{k^{3}}∼Bk^{-\lambda }$$ (28)

In Eq (28), *k* represents the quantity of neighbors, and *B* represents the simplification of 2*m*^2^*t*/(*m*_0_+*t*) in Eq (28), where *m*_*0*_, *m* and *t* represents the initial setting node number, the connecting node number for each adding node and the number of adding times, respectively.

Under this assumption, the degree of each node can be shown as the probability sum: *k*_*i*_ = ∑_*k*_*P*(*k*)∙*k*. In this situation, the above Eqs (2), (3) and (5)–(8) can be transformed as:

$$T(n)=\sum_{i}^{n}k_{i}/n=\sum_{i}^{n}\sum_{k}P(k)∙k/n$$ (29)

$$H_{j}(n)=\sum_{i}^{n}{a_{ij}∙k}_{i}/T=\sum_{i}^{n}a_{ij}∙\sum_{k}P(k)∙k/n$$ (30)

$$TI=\sum_{j}^{m}\sum_{i}^{n}|a_{ij}|∙k_{i}/m=\sum_{j}^{m}\sum_{i}^{n}|a_{ij}|∙\sum_{k}P(k)∙k/m$$ (31)

$$HI_{j}=\sum_{i}^{n}{|a}_{ij}|∙k_{i}/TI=\sum_{i}^{n}{|a}_{ij}|∙\sum_{k}P(k)∙k/TI$$ (32)

What is different is that in this case the simplify assumption cannot be done $\sum_{k}P(k)∙k=\bar{k}$ as before. Eqs (10)–(12) can be rewritten as:

$$\frac{ds_{k}(t)}{dt}=-\alpha s_{k}(t)\sum_{k^{\prime }}P(k^{\prime })i_{k^{\prime }}(t)-\gamma s_{k}(t)\sum_{k^{\prime }}P(k^{\prime })r_{k^{\prime }}(t)$$ (33)

$$\frac{di_{k}(t)}{dt}=\alpha i_{k}(t)\sum_{k^{\prime }}P(k^{\prime })s_{k^{\prime }}(t)-\beta i_{k}(t)\sum_{k^{\prime }}P(k^{\prime })r_{k^{\prime }}(t)-\eta i_{k}(t)$$ (34)

$$\frac{dr_{k}(t)}{dt}=\gamma r_{k}(t)\sum_{k^{\prime }}P(k^{\prime })s_{k^{\prime }}(t)+\beta r_{k}(t)\sum_{k^{\prime }}P(k^{\prime })i_{k^{\prime }}(t)+\eta i_{k}(t)$$ (35)

where *s*_*k*_(*t*)+*i*_*k*_(*t*)+*r*_*k*_(*t*) = 1 and *s*(*t*) = ∑_*k*_*P*(*k*)*s*_*k*_(*t*), *i*(*t*) = ∑_*k*_*P*(*k*)*i*_*k*_(*t*), *r*(*t*) = ∑_*k*_*P*(*k*)*r*_*k*_(*t*). In the following section simulation method will be used to see the evolution in global situation.

RETRACTED

In conclusion, in uniform network, larger *n* and *u* are good for information spreading when *i*_*j*_ and *r*_*j*_ do not change, because it leads to larger *J* and make the transformations among these groups easier. Besides, for real networks the larger *n* will lead to more complex cases, the global results will be different from the local analysis. The value of *u* is changing all the time during the information spreading process, and the first coming information will meet very high *u*, while the later one will meet lower *u*. In BA network, the transform dynamic equations are expressed at different degree *k* levels. Since *J* is only based on the local information, numerical simulation is also needed to analyze the global spreading nature with different system parameters.

## 4. The simulation results and analysis

### 4.1 Presentation of simulation methods and initial setting

In this section, simulation method is used to analyze this multi-information propagation system from global spreading process. The simulations will be separated into two large parts by different network structure: the uniform network and the non-uniform network (here BA network is used). Since the multi-information system here is a nonlinear system, to exclude the effect of initial setting, the largest degree level of top 5% is set to be group *S* rather than group *I* or *R* in non-uniform system, while in uniform system, the initial group distribution is totally random.

For each case, the initial distribution is initialized by 5 different random seeding to avoid the initial setting influence, and each initialized distribution will be averaged by 10 independent simulations separately to avoid the processing disturbance. The final output is the average result of these 50 independent simulation results.

RETRACTED

Since system here is a multi-information spreading system, here the rule is illustrated for selecting information. It is supposed there are *m* pieces of information in this system, and the simulation time is also separated into *m* parts. Each time zone is set as unit time length. The information selecting probability (probability density function) is Gaussian distribution with its mean value changing continuously when the simulation time is going on, and the standard deviation of this Gaussian distribution is 0.5. It is supposed that there are 5 different pieces of information in this simulation system labeled as 0, 1, 2, 3, 4, respectively. 5 pieces of information are set because fewer pieces of information may miss the differences among different information and much more information will waste the computer resource. The initial mean value of this probability density function is 0, with the simulation time going on, it increases continuously and the final value is 5. The mean of this probability distribution function will increase and the form of this probability distribution remains the same. At each simulation step, the system generates a random number under this probability distribution function. This random number will be rounded down to its nearest integer, like 1.4 rounded to 1, and this final integer number is the system picking information label. The selecting process is just as Fig 6 shows. Under this rule, it is easily to find that the No. 0 information is the first popular information, which means in the first time No. 0 information is the most possible picked information. With the time going on, the popular center will move to No. 1, 2 and so on, respectively. In this way, it is available to highlight the different popular information in different time. Besides, the choose of node is totally random, each node can be selected with equal probability.

**Fig 6:** The diagram of information pick mode.

Since at each step, the selected node needs choosing one of its neighbors to determine the judgement *J*, here the pick probability are set to equal to each neighbor’s degree over the sum of all neighbors’ degree:

$$P_{pick}(c_{B})=d_{c_{B}}/\sum_{i}^{n}d_{i}$$ (36)

where *P*_*pick*_(*c*_*B*_) represents the pick probability of neighbor node *c*_*B*_.

In the following simulations, the basic benchmark parameters setting are α_0_ = 0.40, β_0_ = −0.80, γ_0_ = −0.80, η_0_ = −0.80. The system size is set as *N =* 1000, and the initial group setting proportion is *S*: *I*: *R* = 0.90: 0.05: 0.05. Since the occupancy of group *I* is the focus of this study, the peak value of group *I* will be particularly picked during the spreading process to analyze.

RETRACTED

### 4.2 Uniform network simulations and analysis

In uniform network, based on the benchmark initial setting, the influences from different neighbor number *n* are checked first (Fig 7(A)). It can be seen that the *I* peak value (*I*_*max*_) of No. 0 and 1 information always stay on the top, while the last label, No. 4, information is always stay at the bottom. The information between them encounter large fluctuation. It can be seen that both information No. 2 and 3 have very low *I*_*max*_ when *n* is small (*n* = 4, 5), and then increase sharply when *n* = 6. After that No. 2 information stays on the top with oscillation, while No. 3 information drops sharply (*n* = 7), then stays at the bottom and never increases anymore. Besides, with the increase of *n*, the No. 2 information appears an obvious drop when *n* > 16 with large mean standard derivation (MSD). In section 3 the uniform network situation is analyzed in detail, and now the exact numerical results can be calculated with given detail parameters.

**Fig 7:** (a) the evolution tendency of each information’s *I*_max_ with different neighbor number *n*. (b) the minimum necessary number of *I* node among neighbors when No.2 information can successfully spread. (c) the total spreading probability of No.2 information with initial parameter setting for different neighbor number. (d) the modified spreading probability (the total spreading probability multiply neighbor number) of No.2 information with benchmark initial parameter setting for each node in different neighbor number.

The most interesting and most need special analysis evolution is No.2 information evolution. Its change tendency can be explained by the following theoretical analysis. According to Eqs (9) and (23), the minimum of *i* in initial setting is:

$$J_{2}=\tanh\left({n∙i}_{min}\right)\tanh\left(\frac{5i_{min}}{2+i_{min}}\right)\geq \alpha_{0}=0.40$$ (37)

where *i*_*min*_ means the minimum proportion of *I* among neighbors and in that case the *R* group does not exist. The number 2 in the second part of Eq (37) is derived from simulation results that before No. 2 information start to be popular, the No. 0 and 1 information have already reached the peak. For each *n* range from 2 to 20, it is easily to get the minimum number of *I*, the results are as Fig 7(B) shows.

Then the situation is analyzed including *R* group. In the initial group setting, the proportion is *S*: *I*: *R* = 0.90: 0.05: 0.05, so the possibility for each node can transform to group *I* under initial situation is:

$$P(n)=\sum_{{x=n∙i}_{min}}^{n}{[C}_{n}^{x}∙{\left(0.90\right)}^{n-x}∙\sum_{y=0}^{\frac{x-{n∙i}_{min}}{2}}C_{x}^{y}{∙(0.05)}^{y}∙{\left(0.05\right)}^{x-y}]$$ (38)

where (*x*−*n*∙*i*_*min*_)/2 round down to the nearest integer. The results are shown in Fig 7(C). The theoretical tendency is similar to the simulation output, especially in some important turning points. When *n* = 4, the theoretical spreading probability sharply decreases from the top, while the simulation *I*_*max*_ also decreases sharply. In the range *n*∈[10, 16], the *I*_*max*_ of simulation results increases with oscillation on the top, and the theoretical results are also on a continuously increase stage.

RETRACTED

Since the above calculation only consider the probability of single node transformation to *I* from the initial setting, while the structure of network, the connectivity of network is also important in the spreading process. So, the probability *P*(*n*) is multiplied by the neighbor number *n* to approximatively represent the spreading intensity, the results are as Fig 7(D) shows. A horizontal line at *n* = 5 is drawn, the case above this line can get a relatively high *I*_*max*_, while below it the system can only reach a relatively low *I*_*max*_ value except the case when *n* > 16 which have a large MSD. This spreading intensity can partly explain the simulation output, because this theoretical analysis is only based on the initial setting, and it will be more complex with the developing of multi-information spreading.

In order to analyze the different influence from these transformation factors, these 4 parameters from 0.30 to 0.90 (-0.30 to -0.90) are traversed based on the benchmark setting to see the *I*_*max*_ evolution tendency, just as the Figs 8 and 9 shows. Here two different neighbor number cases *n* = 6 and 10 are picked, in *n* = 6 situation almost all the information can reach the top *I*_*max*_ value except the last information, while in *n* = 10 situation the No. 2 information drops a little with large MSD, in the meanwhile the other 4 pieces of information are separated into two totally different parts: No. 0 and 1 information can widely spread with high *I*_*max*_ value, while No. 3 and 4 information cannot spread anymore with very low *I*_*max*_ value. Moreover, for larger *n*, the MSD of middle popular information, such as No.2 information, will be larger, which is unsuitable for simulation analysis.

**Fig 8:** (a)–(d) shows the mean *I*_*max*_ changing tendency in uniform network with the alteration of parameter α_0_, β_0_, γ_0_, *η*_0_, respectively based on benchmark setting for different information. Here the neighbor’s number is *n* = 6.

RETRACTED

**Fig 9:** (a)–(d) shows the mean *I*_*max*_ changing tendency in uniform network with the alteration of parameter α_0_, β_0_, γ_0_, *η*_0_, respectively based on benchmark setting for different information. Here the neighbor’s number is *n* = 10.

The changing tendency from *n* = 6 and 10 are shown in Figs 8 and 9 respectively. From these results, it can be seen that the large changes of *I*_*max*_ for the information are from the alter of α_0_ and γ_0_. The other two parameters, β_0_ and η_0_, do not make large changes in information spreading pattern.

When *n* = 6, with the increase of α_0_, it can be seen that the *I*_*max*_ of these information from later popular to earlier popular drop from the top sharply one by one, until all the information cannot rise anymore. The last popular information is most sensitive to α_0_, while the first popular information can still widely spread even though α_0_ = 0.70. The case of information sensitive to α_0_ can be explained by simply calculation similar to Eqs (37) and (38), and the spreading process phase transformation point of different information from first to last popular information is α_0_ = 0.72, 0.58, 0.46, 0.40, 0.34, respectively (Fig 8(A)). However, with the increase of γ_0_, all the information decreases in a smoother way. The interesting thing is that the falling down timing is different from the situation in α_0_ changing cases: on the falling down stage, the falling down timing is No. 0>No. 1≈No. 2>No. 3, in other words the No. 0 information is the first to fall down even though γ_0_ = −0.74 (Fig 8(C)). This can be explained by theoretical results: the larger *u*, which means the popular of information is easier, can lead to larger judgement parameter *J*, meaning that the transformation from *S* to *R* can be easier to across high γ_0_ limitation. With the continuously increase of γ_0_ limitation, the later popular information starts to fall down one by one with different *u* nature. When this limitation is close to the limitation of transformation from *S* to *I* (where α_0_ = 0.40), the relationship between these two transformation processes (*S* to *I*, and *S* to *R*) becomes competition, resulting in the final output stays around *I*_*max*_ = 0.50. Besides, the alter of β_0_ and η_0_ do not change the nature of information spreading (Fig 8(B) and 8(D)), this is because the transform from *I* to *R* needs many *R* around the node, since the initial setting of *R* proportion is 0.05, so it is hard to complete this process.

The case *n* = 10 gets the similar results comparing to the situation *n* = 6. Since the information sensitive to α_0_ does not change, the phase transformation points move forward a bit (Fig 9(A)), where the later popular information needs lower limitation comparing to the case *n* = 6. The change tendency of *I*_*max*_ with the alter of γ_0_ is also a little different from the case *n =* 6, since with *n* = 10 only No. 0 and 1 information can be in widely spreading, but in very low γ_0_ limitation situation, the *I*_*max*_ of all information will still drop to a very low value (Fig 9(C)). Besides, with the change of β_0_, γ_0_, *η*_0_, it can be seen that the oscillation of *I*_*max*_ for No. 2 information is very large (also with very large MSD, but not drawn in figure), means that the middle popular information will meet lots of uncertainty, the final result for this information will be largely depend on the initial distribution and group transformation process, which will be very hard to forecast the following evolution.

RETRACTED

Based on the benchmark setting, Fig 10 shows the evolutions of individual information from the same initial group distribution with γ_0_ = −0.42, *n* = 10. It can be seen that even from the same initial setting and group distribution, with the developing of information spreading, the differences among these outputs are large. Information No. 0 is the first popular one, the *I* rises first and then falls down to a very low value, except one case still stays on a relatively high value (Fig 10(A)), while for *R* group the percent increases monotonically and then stay on the top value with no change anymore (Fig 10(D)). For No. 2 information, it can be clearly seen that the divergence between low and high *I* situation: in some of cases *I*_*max*_ can be large and stays on the top, while for others *I*_*max*_ can only be very small (Fig 9(B)), but what is different from No. 0 information is that even *I* cannot spread widely, the occupancy of group *R* is still very low (Fig 10(E)). For the last popular information, the *I* and *R* do not increase much (Fig 10(C) and 10(F)).

**Fig 10:** Starting from the same initial setting and group distribution, and based on benchmark setting but with γ_0_ = −0.42, *n* = 10. (a)–(c) shows 10 individual evolutions and also the average change tendency of *I* percent for information No. 0, 2, 4, respectively, while (d)–(f) shows the corresponding results to (a)–(c) for *R* percent evolution, respectively.

### 4.3 Scale-free network simulations and analysis

In the following we analyze the multi-information spreading system in scale-free, or says BA network. The parameter setting is the same with the uniform network case, and we set the initial BA network parameter *m*_*0*_ *= m =* 3.

RETRACTED

Similar to the analysis in uniform network, based on the benchmark setting, the *I*_*max*_ change tendency is presented in BA network with the variation of parameter α_0_, β_0_, γ_0_, *η*_0_, respectively (Fig 11). In many situations, like Fig 11(B) and 11(D), the No.2 information stays in the middle *I*_*max*_ value but with large MSD (not shown). These situations are usually including both two statements: high *I*_*max*_ value and low *I*_*max*_ value, just as the Fig 9(B) shown.

**Fig 11:** (a)–(d) shows the mean *I*_*max*_ changing tendency in BA network with the alteration of parameter α_0_, β_0_, γ_0_, *η*_0_, respectively based on benchmark setting for different information.

In general, the results are similar to those in uniform network but exist some differences. With the increase of α_0_, the decrease of *I*_*max*_ for each information seems to be not so sharply but more smoothly with oscillation (Fig 11(A)). The mix of different degree nodes make the nature of spreading system in larger uncertainty and noise. For the decrease of γ_0_ limitation, it can be seen that the falling down of No. 0 information is still easier than No. 1 information, and the changing tendency extends to a low value almost in a linear way (Fig 11(C)), which is similar to the rule in uniform network (Fig 8(C)). Besides, the change of β_0_ and η_0_ still do not mainly change the spreading nature of this information system, and the oscillations of No. 2 and 3 information are also large.

Since in BA network, the degree distribution is as Eq (28) shows, whether the final states in different degree levels are the same is worth studying. Fig 12 shows the evolution of *S* and *I*’s average occupancy degree level of top 5%, middle 5% and last 5% part, respectively. As seen in different degree level, although the main spreading nature for different degree levels are similar, the change of larger degree level seems smaller. This is because in BA network, the large degree node is surrounded by many different degree nodes, and most of them are small degree nodes, the interaction among them will finally make these different degree nodes be in the similar state. Since the state of small degree node is easier to change, resulting in the state transformation is usually first happened among small degree nodes. Besides, in some situations, lots of changed small degree nodes may still cannot change the state of large degree nodes. So, considering all of these factors above, the final phenomenon should like Fig 12(A)–12(F): the change of smaller degree level seems larger, but the evolution tendencies from all the different degree levels are still very similar.

RETRACTED

**Fig 12:** (a)–(c) shows the average simulation results based on benchmark setting for *S* occupation percentage evolution with each information of the part of degree rank top 5% (0–5%), middle part (47.5–52.5%), last 5% (95–100%), respectively; (d)–(f) shows the *I* occupation percentage evolution corresponding to (a)–(c), respectively.

In summary, in uniform network, it is found that the change of *n* influences the middle popular information most, whose *I* peak value *I*_*max*_ changes largely when *n* changes. In addition, the early popular information always keeps high *I*_*max*_ value, while for later popular information, *I*_*max*_ can only stay at the bottom. It is found that α_0_ and γ_0_ play an important role in this spreading system. With the increase of α_0_, the *I*_*max*_ of the information drops sharply one by one from the last popular information to the first popular information, and all the information are very sensitive to the change of α_0_. With the increase of γ_0_, the *I*_*max*_ of the information falls down one by one from the first popular information to the last popular information, the information reaction order of which is different from that of α_0_. The other two parameters, β_0_ and *η*_0_, have little impact on the spreading system. In BA network, the simulation results are similar to those in uniform network, but the evolution tendencies become smoother due to the mixture of different degree nodes in the system. Besides, in BA network there is no big difference between the evolution tendencies of the information at different degree levels, the only difference is that the change of larger degree level seems smaller. This is because the mixture of different degree nodes makes the small degree nodes can be largely influenced by large degree nodes, while in some situations large amount of changed small degree nodes may still cannot change the state of large degree nodes, leading to all the degree level nodes turning into the similar state but the small degree nodes with larger change.

## 5. Conclusion

A new information transmitting model is adopted to keep users free of disturbing information so that they can focus on the useful ones filtered from the information mass, under the information explosion era. The model is built based on the Susceptible Infected Recovered (SIR) model, with ability of thinking the partial information environment and limiting attention of users. Besides, heat and prevalence are adopted to measure the conversion of situation of nodes. Results of experiment show that the node of the first hot news is easier to converse, for the first hot news gets more attention than the other information. Numerical simulations are conducted to verify theoretical results in both uniform network and BA network. The simulation results show that the early popular information is less vulnerable to the increase of the information acceptance threshold than the later popular information, but the early information is more sensitive to the increase of the threshold of *S* to *R* transformation than the later one in uniform network. While in BA network, the evolution tendencies are similar but smoother than those in uniform network due to the mixture of different degree nodes in the system, and the change tendencies of different degree levels are very similar. The simulations confirm the theoretical analysis results, and it can explain why the first popular information can be the top hot topic for a long time, while the following popular information reach the same high level will be harder even it has the same influence power. In this model, the node state transformation is not determined by initial setting fixed probability as in other research but by people’s limited attention and the local information environment, which is more in line with the information propagation in the real world. This study provides a new perspective for related work. However, there are also some aspects needs to be improved. The interaction among information with different influence power, and the relationship between different information (mutual enhancement, mutual inhibition and so on) should also be considered. In the practical situation of hot news, parts of users can buy the nodes to broaden the information pushing and draw other users’ attention by obligatory pushing the news to the top. This kind of uncertainty cannot be estimated through a fixed model, which is one of the limits of this experiment. Besides, open network can also be considered, which is closer to the real world. These factors will be analyzed in the following papers. Last but not least, several online information platforms with mutual effects as well as human factors should be considered in the after experiments to make the research method reasonable and serious.

RETRACTED

## Supporting information

S1 Dataset The dataset of each simulation result for all the uniform network used in this paper. (ZIP)

S2 Dataset The dataset of each simulation result for all the scale-free network used in this paper. (ZIP)
